# An End-to-End Cardiac Arrhythmia Recognition Method with an Effective DenseNet Model on Imbalanced Datasets Using ECG Signal

**DOI:** 10.1155/2022/9475162

**Published:** 2022-09-29

**Authors:** Hadaate Ullah, Md Belal Bin Heyat, Faijan Akhtar, Sumbul, Abdullah Y. Muaad, Md. Sajjatul Islam, Zia Abbas, Taisong Pan, Min Gao, Yuan Lin, Dakun Lai

**Affiliations:** ^1^State Key Laboratory of Electronic Thin Films and Integrated Devices, School of Materials and Energy, University of Electronic Science and Technology of China, Chengdu 610054, Sichuan, China; ^2^IoT Research Center, College of Computer Science and Software Engineering, Shenzhen University, Shenzhen 518060, Guangdong, China; ^3^Centre for VLSI and Embedded System Technologies, International Institute of Information Technology, Hyderabad 500032, Telangana, India; ^4^Department of Science and Engineering, Novel Global Community Educational Foundation, Hebersham 2770, NSW, Australia; ^5^School of Computer Science and Engineering, University of Electronic Science and Technology of China, Chengdu 610054, Sichuan, China; ^6^Department of Ilmul Qabalat wa Amraze Niswan (Gynecology and Obstetrics), National Institute of Unani Medicine, Rajiv Gandhi University of Health Sciences, Ministry of Ayush, Bengaluru, Karnataka, India; ^7^IT Department, Sana'a Community College, Sana'a 5695, Yemen; ^8^College of Computer Science, Data Intelligence and Computing Art Lab, Sichuan University, Chengdu 610065, China; ^9^Medico-Engineering Corporation on Applied Medicine Research Center, University of Electronic Science and Technology of China, Chengdu 610054, Sichuan, China; ^10^Biomedical Imaging and Electrophysiology Laboratory, School of Electronic Science and Engineering, University of Electronic Science and Technology of China, Chengdu 610054, Sichuan, China

## Abstract

Electrocardiography (ECG) is a well-known noninvasive technique in medical science that provides information about the heart's rhythm and current conditions. Automatic ECG arrhythmia diagnosis relieves doctors' workload and improves diagnosis effectiveness and efficiency. This study proposes an automatic end-to-end 2D CNN (two-dimensional convolution neural networks) deep learning method with an effective DenseNet model for addressing arrhythmias recognition. To begin, the proposed model is trained and evaluated on the 97720 and 141404 beat images extracted from the Massachusetts Institute of Technology-Beth Israel Hospital (MIT-BIH) arrhythmia and St. Petersburg Institute of Cardiological Technics (INCART) datasets (both are imbalanced class datasets) using a stratified 5-fold evaluation strategy. The data is classified into four groups: N (normal), V (ventricular ectopic), S (supraventricular ectopic), and F (fusion), based on the Association for the Advancement of Medical Instrumentation® (AAMI). The experimental results show that the proposed model outperforms state-of-the-art models for recognizing arrhythmias, with the accuracy of 99.80% and 99.63%, precision of 98.34% and 98.94%, and *F*_1-score_ of 98.91% and 98.91% on the MIT-BIH arrhythmia and INCART datasets, respectively. Using a transfer learning mechanism, the proposed model is also evaluated with only five individuals of supraventricular MIT-BIH arrhythmia and five individuals of European ST-T datasets (both of which are also class imbalanced) and achieved satisfactory results. So, the proposed model is more generalized and could be a prosperous solution for arrhythmias recognition from class imbalance datasets in real-life applications.

## 1. Introduction

With the advancement of computerized and automatic electrocardiogram (ECG) analysis, it is widely used in detecting and diagnosing heart diseases, assisting cardiologists with long-term ECG recordings and analysis. One significant indicator of heart disease is the detection of heartbeats, which is an essential factor in detecting arrhythmias. Arrhythmias are irregularities in heart conduction with electrical impulses, resulting in a disturbance in heart rate (irregular rhythm) [1], which necessitates careful, rapid, and frequent examination. In this case, automatic and computerized systems can be more useful. A traditional automatic arrhythmia recognition system includes (i) preprocessing [2], (ii) features extraction such as beat segmentation [3], QRS complex [4], R-peak or R-R interval [5], wavelet transform (WT) [5], time-frequency [6], morphological learning [6], and (iii) classification such as artificial neural network (ANN) [7], support vector machine (SVM) [8], decision tree (DT) [9, 10], and random forest (RF) [8] steps. However, despite a good number of shallow learning methods (features engineering techniques) with promising results for identifying arrhythmias from ECG signals, these are unable to properly describe the optimal features of signals and are prone to overfitting [11]. Furthermore, dealing with unbalanced data while yielding satisfactory results remains difficult [12]. Several researchers attempted to solve these problems by optimizing classifiers' generalization capabilities [13]. Due to the limited nonlinear fitting, the learning parameters in machine learning face a challenge during training to extract all features from ECG. As a result, the pattern recognition performance of classifiers in traditional methods from ECG signals is typically insufficient in the context of big data-driven [14]. Considering the aforementioned challenges of machine learning approaches [15, 16], an effective recognition method that takes a different approach is highly desired in arrhythmia diagnosis.

Deep learning approaches for arrhythmia recognition, such as deep neural networks (DNNs) [17], convolution neural networks (CNNs) [18, 19], recurrent neural networks (RNNs) [18], long short-term memory (LSTM) [20], and combining of these approaches [21], have recently gained popularity [22, 23]. Aside from arrhythmia recognition, deep learning approaches have received a lot of attention recently in other applications, such as emotion recognition from electroencephalography (EEG) [24–28]. Although high-level features learned from ECG inputs of such developed deep learning models automatically perform feature extraction and recognition, satisfactory performance of arrhythmia diagnosis remains a challenge. The major factors behind this challenge are as follows: (i) some patterns of ECG are hard to detect in deep learning because of extensive volume of data demanding for training the deep networks with the target domain, even it is hard to recognize by experienced physicians [17] in some cases, and (ii) deep networks tends to vanishing gradient problems during training. The first challenge could be addressed by a mechanism known as “transfer learning,” in which experienced learning from the upstream dataset (large volume dataset) is transferred into the downstream dataset (target dataset), and pretrained weights from the upstream dataset are used as the target dataset's initial weights [29]. This mechanism could easily solve the deep network overfitting problem. A few contributions to the literature address the transfer learning mechanism for detecting abnormalities in ECG signals [30–33]. In this type of approach, there is no requirement to develop a model from scratch.

However, the appearance of ResNet [34] in deep learning marked a turning point in CNN models. ResNet's interesting developments include shortcut and skip connections between the front and back layers, which aid in resolving vanishing gradient problems. Following the benefits of ResNet, DenseNet [35] introduces an intriguing connectivity pattern among the layers known as “dense connections” for the further improvement of ResNet, in which feature maps for each layer in a dense block are followed by all of its previous layers, with direct connections from low- to high-level layers. As a result, the second challenge of recognizing arrhythmias with satisfactory results could be overcome by developing a model based on the dense connections mechanism. In this study, an end-to-end 2D CNN method with an effective DenseNet model was proposed to recognize arrhythmias from ECG automatically, taking into account the potential benefits of a CNN-based DenseNet model addressing the aforementioned challenge in cardiac arrhythmia recognition. Recently, 2D CNN approaches for arrhythmias recognition have gained popularity because of the transformation of sequential data of beats into their corresponding beat images, which alleviates the time strict alignment problem of beats ignoring the score of fiducial points. The duration and amplitude of various waves of an ECG signal, such as RR intervals, QRS complex, P-wave, and T-wave, are highly sensitive to its dynamic and morphology features. ECG signals from time series data could be transformed into 2D images in a variety of ways, such as time-frequency (short-time Fourier transform (STFT) [36], continuous wavelet transform (CWT) [37, 38], discrete wavelet transform (DWT)), frequency spectrum, own developed python module [39].

Besides, some interesting contributions are introduced in the literature addressing dense connections mechanism for ECG classifications. Rubin et al. [40] proposed a densely connected CNN for atrial fibrillation (AF) detection from ECG by combining the SQI (signal quality index) algorithm to assess the noisy instances in ECG. Importantly, this work discussed an additional challenge of the imbalance problem in private or publicly available arrhythmia datasets, which may significantly impact the accuracy of arrhythmia diagnosis in real-life applications. Importantly, this work discussed an additional challenge of the imbalance problem in private or publicly available arrhythmia datasets, which may significantly impact the accuracy of arrhythmia diagnosis in real-life applications. Some interesting contributions have been demonstrated in the literature for resolving the challenge [12, 41–43]. We have used the weighted categorical cost function [44] to handle the imbalanced data in this study due to the function's several advantages. In this study, a novel and end-to-end 2D CNN-based deep learning method is proposed for cardiac arrhythmia recognition with improved performance, taking into account the aforementioned challenges and opportunities. The following are the key contributions near the end:

- A 2D CNN model is developed to recognize arrhythmias with greater accuracy than state-of-the-art models on imbalanced datasets.
- The proposed model expresses model generalization because it was tested on four datasets without changing any hyperparameters, and the model architecture and results are consistent.
- This achievement is due to the use of some diverse regularization strategies: batch normalization (BN) [45], call-back features [46], weighted random sampler [47], Adam optimizer [48], on-the-fly augmentation [49], and appropriate initialization of layers [50] of the model in the method.

The rest of the paper is expressed as follows. The proposed methodology is presented in Section 2 with details. Results and discussions with study limitations and prospects are included in Section 3. Finally, Section 4 concludes the study.

## 2. Methods and Materials

### 2.1. Dataset Description

#### 2.1.1. MIT-BIH Arrhythmia Database

MIT-BIH arrhythmia database: The MIT-BIH arrhythmia database is a widely used benchmark database for evaluating the performance of arrhythmia detectors. It contains 48 records from 47 subjects (25 males aged 32 to 89 and 22 females aged 23 to 89) with 30-minute two-channel ambulatory Holter ECG recordings. The recordings are sampled at 360 Hz per channel with an 11-bit resolution over a 10 mV range. Its first channel describes the upper signal, MLII (a modified limb lead II), and its second channel describes the lower signal, modified lead V1 (rarely as V2 or V5, and only once as V4), with electrodes placed on the chest in both cases. In the upper signal, normal QRS complexes are more visible. As a result, the upper signal lead is chosen in our study. Records 102 and 104 are involved with patient surgical dressings and records 102, 104, 107, and 217 are involved with paced beats, so we excluded these records from our experiment.

#### 2.1.2. INCART 12-Lead Arrhythmia Database

INCART contains a total of 75 annotated records extracted from the 32 Holter recordings. Every record is thirty minutes long, holds the twelve standard leads, and is sampled at 257 Hz with varying gains from 250 to 1100 per mV. The records were accumulated from the patients who were undergoing tests on coronary artery diseases. Most of them had ventricular ectopic beats, and nobody had pacemakers. ECGs from subjects with arrhythmias, coronary artery disease, ischemia, and conduction abnormalities were preferred for incorporation into the database. Leads II and V1 are two of the 12 standard leads that appear more frequently in this dataset. In the lead II, QRS complexes are more noticeable. As a result, lead II is chosen in this study, similar to the MIT-BIH arrhythmia database. The dataset is used in this study to test the generalization of the proposed model.

#### 2.1.3. MIT-BIH Supraventricular Arrhythmia Database

This database contains 78 two-lead ECG recordings with a sampling rate of 128 Hz, each with half an hour. The annotation of recordings was performed with the Marquette Electronics 8000 Holter scanner firstly, and it was corrected and reviewed later with a medical student. The original labeling was modified in accordance with AAMI recommendations. It is a supplementary dataset of MIT-BIH arrhythmia that is chosen only for testing or evaluating the performance of the proposed model in this study. Only five records, 800, 828, 849, 867, and 873, are considered for transfer learning, and one record, 873, is considered for testing the performance of the proposed model.

#### 2.1.4. European ST-T Database

The database includes 79 patients' ambulatory ECG recordings from 90 annotated snippets. There were 8 women and 70 males, aged 55 to 84, in the study. Each two-hour record includes two lead signals sampled at 250 samples per second with 12-bit resolution across a nominal 20-millivolt input range. After digitization, the sample values were rescaled with reference to calibration signals in the original analog recordings to ensure a uniform scale of 200 analog-to-digital-converter units per millivolt for all signals. Each record is documented by concise clinical reports. These reports, which are stored in the header (.hea) files associated with each recording, summarize pathology, medications, electrolyte imbalance, and technical information. Two cardiologists annotated each record beat by beat, looking for changes in ST segment and T-wave morphology, rhythm, and signal quality. ST segment and T-wave changes in both leads were identified (using predefined criteria that were applied consistently in all cases), and their onsets, extrema, and ends were annotated. Only five records, e0103, e0121, e0202, e0413, and e0614, are considered for transfer learning, and one record, e0121, is considered for testing the performance of the proposed model.

### 2.2. Method Overview

Herein, an arrhythmia recognition framework is made. To begin, annotated data from the MIT-BIH arrhythmia, St. Petersburg INCART 12-lead, MIT-BIH supraventricular arrhythmia, and European ST-T database datasets are selected to categorize the arrhythmias into four classes of interest. The raw data instances are then segmented into available beats and transformed into RGB (Red, Green, and Blue) images via the preprocessing step. The proposed method makes use of the transformed images as input. This framework's model architecture is based on the structure (DenseNet) in [35] to perform recognition. Three dense blocks are created in this model, each with five inner layers, followed by a transition layer to extract the features from our preprocessed images. Finally, preprocessed images are classified as N, S, V, and F (based on AAMI) with two fully connected (FC) layers and a softmax classifier. Based on AAMI recommendations, the class mappings of all datasets are as follows: (1) N-normal, (2) V-ventricular ectopic, (3) S-supraventricular ectopic, (4) F-fusion, and (5) Q-unknown. Because of the involvement of paced and unclassified beats, the *Q* class is not considered in this study. The overall method includes three subsections: (1) data preprocessing, (2) feature extraction and recognition based on the proposed DenseNet model, and (3) model evaluation. We have evaluated the proposed method with the strategies (experiments): *E*_1_-experiment 1 (5-fold stratified cross-validation (CV) on MIT-BIH dataset), *E*_2_-experiment 2 (5-fold stratified CV on INCART dataset, for the generalization purpose of the proposed model), *E*_3_-experiment 3 (MIT-BIH as the training and MIT-BIH supraventricular arrhythmia is only for evaluation), *E*_4_-experiment 4 (INCART as the training and MIT-BIH supraventricular arrhythmia is only for evaluation), *E*_5_-experiment 5 (learned experiences from MIT-BIH arrhythmia dataset by the proposed model are transferred into MIT-BIH supraventricular arrhythmia dataset using transfer learning mechanism), and *E*_6_-experiment 6 (learned experiences from INCART dataset by the proposed model are transferred into MIT-BIH supraventricular arrhythmia dataset), *E*_7_-experiment 7 (MIT-BIH as the training and European ST-T database is only for evaluation), *E*_8_-experiment 8 (INCART as the training and European ST-T database is only for evaluation), *E*_9_-experiment 9 (learned experiences from MIT-BIH arrhythmia dataset by the proposed model are transferred into European ST-T dataset using transfer learning mechanism), and *E*_10_-experiment 10 (learned experiences from INCART dataset by the proposed model are transferred into European ST-T dataset). In the transfer learning mechanism, learned knowledge from a large volume of dataset is transferred into a small volume of dataset (target dataset, which is unseen) during the evaluation. The developed model is fine-tuned in this mechanism by randomly initializing the weights of FC layers remaining the same target classes (N, S, V, and F). Transfer learning is a promising technique for dealing with the challenge of large volume training datasets in deep learning. As a result, the technique is more useful in real-world applications, particularly in remote health monitoring sensor devices. The complete framework with the stratified K-fold cross-validation of the proposed method for *E*_1_, *E*_2_, *E*_3_, *E*_4_, *E*_7_, and *E*_8_ is demonstrated in Figure 1(a). However, the model is in only evaluation mode in the case of *E*_3_, *E*_4_, *E*_7_, and *E*_8_ and tested with the MIT-BIH supraventricular (*E*_3_ and *E*_4_) and European ST-T (*E*_7_ and *E*_8_) datasets.  Figure 1(b) illustrates the workflow of the proposed method using a transfer learning mechanism in the case of *E*_5_, *E*_6_, *E*_9_, and *E*_10_.

### 2.3. Data Preprocessing

Following segmentation, 1D ECG signals are transformed into 2D RGB beat images, fed as input to the developed 2D DenseNet model, segregating various characteristics in the images. Every record in our chosen datasets contains the signals, annotation, and header files for the ECG signals. After downloading the data for each dataset, the annotation file is obtained from these files using Python's Glob module. The individual heartbeats are then segmented from the QRS complexes of ECG signals by slicing each beat using the R-peak wave detection algorithm. This algorithm is more accurate than others in the literature [19]. Once R-peaks are detected, a single beat is traced by taking into account 250 ms (90 sampling points) before and after the R-peak. The distance is sufficient to represent a beat while excluding neighbor heartbeats from an ECG signal [51]. This study's datasets do not all have the same sampling frequency. As a result, the dataset records must be resampled before segmentation. We completed the beats segmentation task using the WFDB Toolbox and the Biosppy Python module at a sampling frequency of 250 Hz. A CSV file of heartbeat sequences for each beat category was received. The Python Matplotlib module and OpenCV are used to convert the segmented beats from the CSV files into their equivalent RGB images of 128128 pixels. Finally, for the four class labels, we received 97720 (N-87311, S-2706, V-7080, and F-623) and 141404 (N-129585, S-1712, V-10001, and F-106) extracted beat images from the MIT-BIH and INCART datasets, respectively. The total of 10244 (N-9797, S-368, V-64, and F-15) and 1673 (N-1622, S-13, V-23, and F-15) beat images for five (800, 828, 849, 867, and 873) records and one (873) record are received from the MIT-BIH supraventricular dataset, respectively. Besides, the European ST-T dataset yielded 44169 (N-43516, S-168, V-364, and F-121) and 10828 (N-10595, S-79, V-91, and F-63) beat images for five (e0103, e0121, e0202, e0413, and e0614) records and one (e0121) record, respectively.  Figure 2(a) shows the segmentation of beats, while Figures 2(b)to 2(f) show the transformed beats images. The transformed images are fed into the developed model for feature extraction. A high-level feature vector is generated from these extracted features, and arrhythmia recognition is performed using a softmax classifier.

### 2.4. Features Extraction Based on Proposed DenseNet and CNN Classifier

Deep learning approaches, particularly several CNNs, have recently emerged as the dominant techniques for image classification [52]. CNNs carry out convolution operations between kernels and tensors. RGB images are used as the input to the developed model. As a result, it should have three channels to represent the intensities of three primary colors (red, green, and blue). The kernels in the convolution operation can be considered as the filters that detect edges, shapes, and other patterns in the input ECG beat images. One major flaw in CNNs is that information may disappear while training the network, a phenomenon known as the “vanishing gradient problem,” as the network's layers become deeper. Though there are several primary approaches to solving the problem, such as layer-wise pretraining and proper activation function selection, dense connections in the DenseNet [35] are a promising mechanism compared to such approaches. DenseNet provided state-of-the-art performance with no degradation despite stacking hundreds of layers. This architecture signifies that the CNNs are deeper and more effective. The DenseNet architecture consists of a series of dense blocks and transition layers [35]. Transition layers facilitate the downsampling, which is required to change the size of features map in CNNs. DenseNet's architecture differs from other CNNs in that it allows for more narrowing layers, which is controlled by a hyperparameter called “growth rate” *k*. Each layer holds a *k* features map at its output. In this study, the minimal optimum configuration consists of three dense blocks, each of which contains five convolutional layers with nonlinear activation functions, ReLUs, and BN, followed by a transition layer, depicted in Figure 3. Each convolutional layer generates 32 feature maps (number of output channels), which are concatenated to all previous convolutional feature maps in the depth direction.  Figure 4 illustrates the concept indicating the reused feature maps from all the preceding layers in a dense block with five layers. For instance, the input channel of the second convolutional layer is 32 (first convolutional layer output), but the input channel of the third convolutional layer is 64 (32^*∗*^2 = 64 for the two prior convolutional layers) and generates 32 output channels, and so on. The produced feature map through the convolving of learnable filters/output channel numbers across the input images is fed to ReLU, a nonlinear activation function. The convolution output channel number as the base value is set to 32. No further significant enhancement is achieved with greater channel numbers, dense blocks, and transition layers. This probably happened due to the small volume of preprocessed images during training the network compared to ImageNet. The convolutional layers are the prime components of CNNs, where major functions of CNNs are performed. Large filter 7 × 7 is considered at the starting of the model in the convolution layer with a spatial downsampling of striding of 2 to conceal the inconsequent features from images. In the preprocessed images, the desired features appear in the narrow part of the full image. And hence, the subsequent convolution layers in the dense blocks with a small size of 3 × 3 and no spatial downsampling are chosen to extract the locally replicated features. As a result, the computational cost of the model is reduced. The employed ReLUs in the dense blocks and transition layers help to suppress vanishing gradient problems during training. BN [45] layers are used to accelerate the training. As a result, the learnable parameters converge with the imminent possible time of training. It also suppresses the sensitivity and interior covariate shift of training in the direction of weight initialization. This is one kind of regularization technique to reduce overfitting during the training phase. The weights during training are made with the gradient-based backpropagation mechanism.

As shown in Figure 3, a transition layer is embodied after each block as the adjacent two blocks that minimize the computational complication with a bottleneck structure. It reduces the dimension of the feature map by removing the learnable parameters. The transition layer receives activations from all of the dense block's preceding kernels. It consolidates them using convolution and pooling operations. Its primary functions are convolution and pooling. Conv., BN, ReLU, and average pooling layers are included in each transition layer. Each transition layer's average pooling layer calculates the average for each patch of feature maps and extracts average spatial high-level features. It also serves as a translation-invariant to help filters and kernels detect the morphological shapes of input images. No learnable parameters are produced from this layer. The output shape of the last pooling layer in the final transition layer is 64 × 16 × 16 with a kernel size of 2 × 2 and stride of 2, as shown in Table 1. The convolutional layer with a 1 × 1 kernel size in the transition layer is used to capture the information across the channel features and deliver the identical output feature maps of 32 in the convolutional layer for the next block, which goes through the average pooling layer with subsampling. The transition layer can also play the compression preface to control the model size by a factor *θ*, called compression in the 0 < *θm* ≤ 1 range. If a dense block has *m* feature maps, the following transition layer produces *θm* output feature maps. In our experiment, we have fixed *θ* = 1 to keep the number of feature maps unchanged across the transition layers. After passing all blocks and transition layers, the feature map of the last average pooling layer is reduced to 64 × 16 × 16, which goes to linear layers for the classification. The output of the linear layer contains the high-level model ascertainment. These layers learn the features vector so that the softmax layer can properly recognize the preprocessed images. The final linear layer's output channel numbers are set to the required number of classes and fed through the softmax activation function for the final predicted labels. In our study, two linear layers are used to ensure that the model learns input patterns correctly. Finally, at the model's end, a softmax layer is included to recognize the arrhythmia labels using numerical processing.

### 2.5. Cost Function and Evaluation Metrics

The cost function or cross-entropy loss is used to assess how well a model is trained. It represents the difference between training samples and predicted labels, thus scoring the training loss. It bridges the gap between measured labels and targets. The function displays the training efficiency of a model. A gradient-descent-based optimizer with a learning rate controls the loss of cost function. Adagrad, Adam, and Adadelta are a few well-known optimizers. Adam optimizer function is used in our experiment, which gets to the optimal points faster than others [48]. This weighted categorical cost function is better suited to dealing with imbalanced data [44, 53]. The MIT-BIH, INCART, MIT-BIH Supraventricular, and European ST-T datasets are more unbalanced. As a result, we chose this function in our study to address the class biasing issue. Let *w* represent the vector weights of the prescribed classes, with a large *w*_*i*_ value corresponding to a high penalty applied to the incorrect label predictions. The weighted categorical cost function is as follows:

(1) $$\begin{array}{c} CE=-\frac{1}{D}\overset{D}{\underset{j}{\sum }}\overset{C}{\underset{i}{\sum }}w_{i}t_{ij}\log p_{ji}. \end{array}$$

where *D* represents the training samples, and *C* narrates the class numbers. As for the example, if *t*_*j*_ holds the class *i*, *t*_*ji*_ = 1 and *p*_*ji*_ will be the predicted probability; otherwise, *t*_*ji*_ = 0.

The performance of our proposed method is evaluated with four metrics: precision, recall, *F*_1-score_, and accuracy, which are expressed in (2) to (5) [54–56], where TP, FP, TN, and FN are the true positive, false positive, true negative, and false negative, respectively. TP represents the beat recognition result in which positive is represented as positive, whereas FN represents the result in which positive is represented as negative. TN, on the other hand, defines the beat identification result in which the negative is evaluated as negative, whereas FP defines the result in which the negative is evaluated as positive. The recall and precision parameters could be used to specify the model's sensitivity and exactness. *F*_1-score_ is used to capture the accuracy by summing up the recall and precision for every predicted class sample. Finally, accuracy assesses the method performance across all beat classes. The metrics equations are as follows:

(2) $$\begin{array}{c} precision=\frac{TP}{TP+FP}. \end{array}$$

(3) $$\begin{array}{c} recall=\frac{TP}{TP+FN}. \end{array}$$

(4) $$\begin{array}{c} F_{1-score}=2\times \frac{precision\times recall}{precision+recall}=\frac{2TP}{2TP+FP+FN}. \end{array}$$

(5) $$\begin{array}{c} Accuracy=\frac{TP+TN}{TP+FP+TN+TF}. \end{array}$$

### 2.6. Experimental Details

All experiments are carried out in PyTorch open-source framework on Windows 10 with Intel Corei5-7400 CPU @ 3.00 GHz, 8 GB RAM, and an NVIDIA GeForce RTX 2070 graphic card with 8 GB memory. For proper initialization, an intelligent weight initialization mechanism for the available layers in the model is required, which aids the model in alleviating biasing. Layer weights could be expressed as kernels and groups of kernels that form a single layer. The proposed model employs the Kaiming normal distribution [50] to initialize the weights in all convolution layers. All BN layers' biases and weights are initialized with the constants 0 and 1, respectively. The Xavier initializer and a constant 0 are used to initialize the weights and biases of fully connected layers, respectively. The primary goal of using these initializers is to balance the gradients scale across all kernels. The performance of a model is highly dependent on the training to testing sets ratio. As a result, the random split technique is used to partition the entire set of preprocessed images into a validation set. The K-fold cross-validation strategy is used to train and evaluate the model. A validation set is typically required to confirm whether or not the model has achieved sufficient accuracy using the training and testing set ratio settings in the training module. Without the validation set, the model could have become overfit. In the hold-out evaluation strategy, K-fold cross-validation is a promising technique for resolving such changing issues as training and testing set ratio. In this strategy, the samples are randomly grouped into the total *k*-fold, and *k* splits are generated. We used stratified 5-fold cross-validation in our study. As a result, in each split, one fold serves as the validation or testing set, while the remaining four folds serve as the training set. In this case, 10% of the total extracted beat images are preserved for testing, while the remaining 90% are used for model training, resulting in a training and testing splitting ratio of 9 : 1.5-folds reducing the computation cost while increasing the likelihood of samples from each class entering each fold. Furthermore, a stratified K-fold ensures that samples from each class enter each fold, reducing the class imbalance problem more effectively than K-fold. The initial learning rate and batch size are set to 0.001 and 32. To optimize the cross-entropy loss, a gradient descent optimizer with a learning rate scheduler is required. In this study, the Adam optimizer [48] with the PyTorch REDUCELRONPLATEAU scheduler is chosen to achieve the desired performance. If the validation loss becomes a plateau for 5 consecutive epochs, the learning rate is reduced by 0.1. During the training process, a weighted random sampler [47] is also used to ensure the representativeness of the equal samples from each class. To achieve the optimal training time, an appealing regularization technique called early stopping [46] is used. If the validation loss remains constant for the next eight epochs, the training is terminated, and the overfitting is reduced. In the training module, the transformed 2D RGB images are simply rotated randomly by 6 degrees before being converted into tensors; this technique is known as “on-the-fly augmentation” of data. This is also a likely factor in reducing model overfitting during training. Finally, the delivered accuracy of our proposed method in *E*_1_ and *E*_2_ on the extracted beat images from the MIT-BIH and INCART arrhythmia datasets is 99.80% and 99.63%, respectively. Furthermore, *E*_3_, *E*_4_, *E*_5_, *E*_6_, *E*_7_, *E*_8_, *E*_9_, and *E*_10_ achieve accuracy of 99.70%, 99.94%, 99.70%, 99.87%, 99.90%, 99.95%, 99.87%, and 99.95%, respectively.

## 3. Results and Discussion

### 3.1. Classification Results

In this study, extracted heartbeat images from ECG signals from four publicly available imbalanced datasets are used to detect arrhythmias in cardiac patients. It is attempted to improve the detection performance by looking into issues where the developed CNN models for arrhythmia recognition are incompetent. A confusion matrix, depicted in Figure 5(a), could express the performance details of all metrics on the MIT-BIH arrhythmia dataset (*E*_1_). The confusion matrix is nonnormalized row-wised. The entries in the diagonal correctly represent beat recognition, while the entries in the off-diagonal express the beat misclassification rate. The rows of Figure 5(a) show that the 87150 N, 7061 V, 2691 S, and 620 F beats are correctly classified out of 87311, 7080, 2706, and 623 beats, respectively. Only 161 N, 19 V, 15 S, and 3 F beats are incorrectly classified. Despite class imbalance issues in the MIT-BIH arrhythmia dataset, it indicates the intended accuracy in each class. The overall accuracy, *F*_1-score_, recall, and precision achieved in standard testing are 0.9980, 0.9891, 0.9996, and 0.9834, respectively.  Table 2 shows a summary of all metrics (average accuracy, precision, recall, and *F*_1-score_) from the confusion matrix (shown in Figure 5(a)) received in *E*_1_. This table clearly shows that the average values for all metrics are close to the overall values, indicating that the developed training module for testing the experiments has generalized. The average accuracy, *F*_1-score_, recall, and precision achieved are 0.9990, 0.9892, 0.9963, and 0.9823. The table also shows that the F beat identification precision is low compared to other beats, resulting in a lower *F*_1_score_.  Figure 5(b) depicts the loss curves used in this experiment for model training and testing. The training loss curve is nearly stable after 61 epochs, whereas the testing loss curve changes abruptly at the start and is nearly stable after 61 epochs, analogous to the training loss curve. The model is halted after 123 epochs due to the use of an early stopping feature during training and evaluation, even though the total number of epochs is set to 200. As a result, the developed model efficiently completes the training and evaluation process without encountering any overfitting issues. In this experiment, the minimum validation loss is 0.0233. Finally, we can say that the model produced the desired level of achievement on our preprocessed images from the MIT-BIH arrhythmia dataset.

A confusion matrix was used to figure out the performance details of all matrices on the INCART arrhythmia dataset (*E*_2_), shown in Figure 6(a). According to the rows of the confusion matrix, the 129124 N, 9964 V, 1685 S, and 106 F beats are correctly classified out of 129585, 10001, 1712, and 106 beats, respectively. Only 461 N, 37 V, and 27 S beats are incorrectly classified; all F beats are correctly classified. It also expresses the desired accuracy in each class despite the INCART dataset's class imbalance issues. The overall accuracy, *F*_1-score_, recall, and precision achieved in standard testing are 0.9963, 0.9891, 0.9942, and 0.9894, respectively.  Table 3 shows a summary of all metrics (average accuracy, precision, recall, and *F*_1-score_) from the confusion matrix (shown in Figure 6(a)) received in *E*_2_. It is also clear from this table that the average values for all metrics are close to the overall values. Average accuracy, *F*_1-score_, recall, and precision obtained are 0.9981, 0.9897, 0.9942, and 0.9854, respectively. The table also shows that the precision for V beat identification is low in comparison to other beats, resulting in a lower *F*_1-score_.  Figure 6(b) depicts the loss curves for the model's training and testing. The training loss curve is nearly stable near 75 epochs, whereas the testing loss curve changes abruptly at the beginning and remains nearly stable after 75 epochs, analogous to the training loss curve. Despite the fact that the epoch is set to 200, the model stops at 193 epochs. The model successfully completes the training and evaluation process with no overfitting issues. In this experiment, the minimum validation loss is 0.0234. As a result, the model achieved the desired level of accuracy on our preprocessed images from the INCART arrhythmia dataset. The delivered results of all the measured matrices and minimum validation loss from both experiments are depicted in Table 4. From Tables 2–4, it is observed that the average and overall values for all measured metrics in both experiments are almost the same despite data and features variability of ECG signals in both datasets (MIT-BIH and INCART). This also indicates the generalization of the proposed model.

The graphs for the three matrices such as accuracy, F_1-score_, and recall in *E*_1_ and *E*_2_, respectively, are shown in Figures 7(a) and 7(b). It is clear from these graphs that the values of these matrices grew as the number of epochs increased and became nearly steady from 61 epochs in *E*_1_ (Figure 7(a)) and 75 epochs in E2 (Figure 7(b)). The initial changes in the graphs are sudden since it takes some time for the testing samples to adapt to the trained model.

The trained model on MIT-BIH in *E*_1_ and INCART in *E*_2_ is also tested in *E*_3_ and *E*_4_, respectively, with MIT-BIH supraventricular. The reached evaluated average values of all performance metrics (average accuracy, precision, recall, and *F*_1-score_) in *E*_3_ and *E*_4_ are figured out by the achieved confusion matrices, demonstrated in Figures 8(a) and 8(b), respectively. A summary of all reached metrics from the confusion matrices depicted in Figures 8(a) and 8(b) is illustrated in Table 5. The obtained average accuracy, *F*_1-score_, recall, and precision from Figure 8(a) are 0.9985, 0.9639, 0.9992, and 0.9375, respectively, whereas from Figure 8(b), the reached average accuracy, *F*_1-score_, recall, and precision are 0.9997, 0.9919, 0.9998, and 0.9844, respectively. The overall achieved accuracy, *F*_1-score_, recall, and precision in *E*_3_ are 0.9970, 0.9639, 0.9992, and 0.9375 respectively, while in *E*_4_, the overall reached accuracy, *F*_1-score_, recall, and precision are 0.9994, 0.9919, 0.9998, and 0.9844, respectively, demonstrated in Table 6. Tables 5 and 6 show that the average and overall values for all measured metrics in both experiments are almost identical, which also expresses the generalization of the proposed model.

The trained model on MIT-BIH (*E*_1_) and INCART (*E*_2_) datasets is scored by *E*_5_ and *E*_6_, respectively, with MIT-BIH supraventricular using a transfer learning mechanism. The reached evaluated average values of all performance metrics (average accuracy, precision, recall, and *F*_1-score_) in *E*_5_ and *E*_6_ could be figured out from the achieved confusion matrices, demonstrated in Figures 9(a) and 9(b), respectively. A summary of all metrics from the confusion matrices depicted in Figures 9(a) and 9(a) is illustrated in Table 7. The average accuracy, *F*_1-score_, recall, and precision in *E*_5_ are 0.9983, 0.9892, 0.9927, and 0.9859, respectively, whereas in *E*_6_, the reached average accuracy, *F*_1-score_, recall, and precision are 0.9994, 0.9955, 0.9970, and 0.9939, respectively. The overall achieved accuracy, *F*_1-score_, recall, and precision in *E*_5_ are 0.9970, 0.9892, 0.9927, and 0.9859, respectively. In contrast, the overall reached accuracy, *F*_1-score_, recall, and precision are 0.9987, 0.9954, 0.9971, and 0.9939, respectively in *E*_6_, demonstrated in Table 8. From Tables 7 and 8, it is also observed that the average and overall values for all measured metrics in both experiments are nearly identical, indicating that the proposed model is generalizable. The loss curves (training and testing) for *E*_5_ are shown in Figure 10(a). The curves are almost stable to 40 epochs. The model is halted at only 72 epochs due to the use of early stopping feature in our developed training and testing module. It is also observed from Figure 10(a) that the developed model completes the training and validation process without facing any overfitting issues with the minimum validation loss of 0.0236. A similar scenario is also observed in Figure 10(b) for *E*_6_, where the loss curves almost remained stable from 60 epochs. The model is halted at 78 epochs with the same minimum validation loss.

The trained model on MIT-BIH in *E*_1_ and INCART in *E*_2_ is evaluated with the European ST-T database in *E*_7_ and *E*_8_, respectively. The achieved confusion matrices, as seen in Table 9, quantify the reached evaluated average values of all performance metrics (average accuracy, precision, recall, and *F*_1-score_) in *E*_7_ and *E*_8_. In *E*_7_, the overall accuracy, *F*_1-score_, recall, and precision are 0.9990, 0.9664, 0.9802, and 0.9523, respectively, whereas in *E*_8_, the overall accuracy, *F*_1-score_, recall, and precision are 0.9995, 0.9802, 0.9865, and 0.9742. Using a transfer learning technique, the trained models on the MIT-BIH (*E*_1_) and INCART (*E*_2_) datasets were further scored by *E*_9_ and *E*_10_ using the European ST-T database, respectively. The achieved confusion matrix, shown in Table 10, could be used to determine the evaluated average values of all performance indicators (average accuracy, precision, recall, and F_1-score_) in *E*_9_ and *E*_10_. When comparing to *E*_9_, the overall attained accuracy, *F*_1-score_, recall, and precision in *E*_9_ are 0.9987, 0.9839, 0.9912, and 0.9733, respectively, while these are 0.9995, 0.9901, 0.9959, and 0.9847 in *E*_10_.  Figure 11(a) depicts the loss curves (training and testing) for *E*_9_. The curves are nearly stable after 40 epochs. Because of the early stopping feature, the model is halted after only 72 epochs. It is also clear from Figure 11(a) that the developed model successfully completes the training and validation processes with a validation loss of 0.0236. A similar scenario is shown in Figure 11(b) for *E*_10_, where the loss curves are nearly stable after 85 epochs and the model is stopped at 78 epochs with the same minimum validation loss.

### 3.2. Discussions

In this section, we will first discuss the issues of why our proposed deep approach provides satisfactory results in arrhythmia recognition. First, deep CNNs have learned the dominant features with their convolution layers, and the outcome is investigated with the resulting classifier. Furthermore, the class activation map from the CNN-based models could be easily reached for the visual analysis compared to RNN and LSTM employed for the sequential modeling. Visual analysis is a significant factor in medical diagnosis. Second, the most crucial stage of the experiment is segmenting and transforming ECG signals into beat images, where R-peak detection or beat segmentation is reached based on a well-known and influential algorithm (Pan-Tompkins) on the arrhythmia datasets. Third, DenseNet architecture has some inspirable benefits compared to other CNN architectures, such as being easy to train by delivering the promoted stream of information, reusing features, fewer parameters to train, and alleviating vanishing gradient problems. Forth, some diverse mechanisms are used such as early stopping [46] and on-the-fly augmentation [49] that help to stop overfitting of the model, weighted random sampler [47] to reduce the class imbalance problem, Adam optimizer [48] to converge the model quickly with the minimum validation loss, and proper initialization of model layers [50]. In addition, data imbalance problems negatively affect the performance of a model. So, in this study, we have used a simple class weighting strategy to resolve the issue of data imbalance. The smaller the class size scores, the more considerable the class weight from the training samples. That class weight is utilized to measure the weighted loss during training so that loss from the smaller class is more significant than the larger class. The strategy is also more apparent from our expressed used loss function in Section 2.5. Previously, some researchers attempted to resolve the class imbalance problem in different ways. Al Rahhal et al. [41] addressed a scenario to handle the data imbalance problem using the focal loss technique [42]. An interesting study by Rajesh and Dhuli [12] with three-level data preprocessing approaches: ROU (random oversampling and undersampling), DBB (distribution-based balancing), and synthetic minority oversampling technique with random undersampling (SMOTE + RU) was observed to handle the data imbalance problem. Our employed cross-entropy loss function can also handle such data imbalance issues. It is demonstrated in [57] that, without using the class weighting strategy, the model's performance is not improved with only focal loss. Moreover, many prior promising models in this sense demand enormous in-depth domain ideas for the preprocessing and feature extraction. On the other hand, our proposed method needs the minimum skill in preprocessing and feature extraction while obtaining better performance even compared to deep learning approaches, as demonstrated in Table 11. The developed model extracts desirable activation on intensity, edge, and shape of the peak of our preprocessed beat images. The background is not so important here because extracted beats appear only in a small portion of the image. The satisfactory performance of the developed model represents the learned features from the images after training. The model is well correlated and embedded with the desired classes concerning the high dimensional (mapped in two dimensions) feature space, which is more evident from the confusion graph and evaluated matrices. So, we are assuming that the averaging procedure of representation performs well. The morphological and dynamic characteristics of all datasets are analogous despite data and features variability of ECG signals, and identical experimental dealing is performed on all datasets. Furthermore, the reached performance results on all datasets with the developed model are almost identical, as illustrated in Tables 2to 10. This expresses the generalization of the developed model.

We have compared our findings with [12, 36–39, 58, 59, 61, 62] in Table 11, where the authors employed almost similar approaches with our works in case of 2D CNN. In the table, we have only placed the results from *E*_1_ and *E*_2_. The results demonstrate that our developed DenseNet outperforms compared to others. It represents the effectiveness of the developed model. *F*_1-score_ is an effective performing metric compared to accuracy on imbalanced datasets, justifying the sensitivity and exactness of a model, where recall and precision are summed up as the harmonic mean. It is observed from the table that the scores of all measured metrics in both experiments on MIT-BIH and INCART datasets, respectively, are almost identical, which indicates the generalization of the proposed method. From Table 11, it is also shown that all 2D CNN approaches deliver better results compared to 1D CNN as well as hand-crafted features engineering techniques. We have also tested our proposed method in 1D CNN form (with time series data) following experiments 1 and 2. The achieved results in both experiments are poor compared to all experiments (*E*_1_–*E*_10_) in 2D CNN. The reached accuracies are 97.56% and 97.65%, respectively, following *E*_1_ and *E*_2_. 1D CNNs are less versatile than 2D CNNs. So, the transformation mechanism of sequential data of beats into their equivalent beat images is a promising strategy. Indeed, it is not practicable to thoroughly compare our study with the previous studies because various strategies are used in the preprocessing stage and model designing. R-R intervals or R-peaks, duration, and amplitude of the QRS complex of ECG are highly sensitive to its dynamic and morphology. The transformation-based method reduces the problem of strict time alignment; it ignores the scoring of fiducial points of heartbeats. The nonlinear and nonstationary characteristics of ECG heartbeats due to the heart's episodic/irregular electrical conduction are the significant factors behind such problems. Moreover, heartbeat-based arrhythmias are classified mainly into two categories, (i) tachycardia and life-threatening ventricular fibrillation that need early diagnosing and treatment with the defibrillator, and (ii) non-life-threatening arrhythmias but require further treatment. AAMI divides non-life-threatening arrhythmias into five classes (N, S, V, F, and Q), where each beat category significantly differs in morphology from others and holds some subclasses with various shapes that introduce a massive challenge for physicians to diagnose manually. The N class includes normal (N), right bundle branch block (RBBB), left bundle branch block (LBBB), atrial escape (e), and nodal (junctional) escape (j) beats; S class includes aberrant atrial premature (a), supraventricular premature (S), nodal (junctional) premature (J), and atrial premature (A) beats; V class includes ventricular escape (E) and premature ventricular contraction-PVC (V) beats; F class only includes the only fusion of normal and ventricular (F) beats; Q class includes paced (/), unclassified (Q), and fusion of normal and paced (f) beats but this class is not considered in our study due to the involvement of paced and unclassified beats. Moreover, an automatic diagnosis with deep learning methods compensates the manual interpretations effectively and efficiently and visual errors of physicians with reduced workloads and medical costs. Our study of automatic arrhythmia recognition is based on AAMI recommendations and provides the desired outcomes. It is observed from the confusion matrix graphs in Figures 5(a), 6(a), 8, and 9 and Tables 9 and 10 that N is more noticeable compared to the remaining beats; again V and S beats are more remarkable than F. It exposes that their ratios are misbalancing, but the proposed method classifies each category properly without biasing towards their majority class.

Experiments 3, 4, 7, and 8 show that the proposed model is only tested with two different unseen datasets (MIT-BIH supraventricular and European ST-T) after training with MIT-BIH and INCART datasets. The outcomes of both experiments are satisfactory, which expresses the model's effectiveness. As a result, the proposed method could prosper in wearable devices such as medical bracelets, wristwatches, and vests for instantaneous cardiac conditions. It could also be a booming approach in telemedicine due to its lightweight compared to fundamental DenseNets (DenseNet-121, DenseNet-169, DenseNet-201, and DenseNet-264) [35]. The lightweight of the proposed model also indicates its more usefulness in storage constraint devices such as mobile, portable/wearable healthcare devices. Transfer learning is becoming popular nowadays due to handling the challenge of huge data demanding for deep model training (the most private and publicly available datasets are currently of small volume). In this approach, the model is not trained from scratch, so it helps to reduce the overfitting problem of a deep model [32] and enhance the computational efficiency. The mechanism could also be a prosperous solution for storage constraint devices in real-life applications. We evaluated our proposed method using this mechanism in experiments 5, 6, 9, and 10. We achieved satisfactory findings by considering only five records/individuals from a different dataset. We have also evaluated the proposed model with ten records/individuals from the same dataset and received almost the same results, which also expresses the model's generalization.

However, there are a few open challenges instead of achieving satisfactory results with our proposed method. First is the intrapatient paradigm in *E*_1_, *E*_2_, *E*_3_, *E*_4_, *E*_7_, and *E*_8_, where the same patient heartbeats are likely to arrive in training and testing sets. This circumstance may lead to biased results. The patient-specific study could be the solution to this challenge. Second, arrhythmia recognition based on a single beat has some limitations to a few extents as the relevant distinction. Short segments from the ECG signals or adaptive beat size length segmentation could be the interpretation of this issue. Third, there is no doubt that it is computationally intensive, so it is more applicable for offline applications in medicals and clinics compared to resource constraint devices. A method's computational efficiency varies with the hardware configuration of the utilized PC. Deep learning-based methods require high computational complexity compared to morphological-based techniques. Hence, these are slower in real-life applications [63]. So, it is suggested that deploying deep learning-based methods in real-life applications where bid data dealing is required is more feasible. Forth is efficiency; it will be hard to deploy our proposed method into portable healthcare devices for real-life applications. In that case, designing the lightweight deep model is directed, or models compression techniques such as weight sharing and knowledge distillation are used. Fifth is integration with expert features; it is hard to integrate a trained deep model with the existing expert features. To handle the issue, domain expert knowledge could be directed to design a deep model. Sixth is noise robustness: a deep method that automatically extracts all features from the signals, including different types of real-world noises, which may lead to incorrect results. So, some researchers tried to resolve the issue by fitting denoising/filtering techniques before commencing data into the input of deep models, but some valuable information could be omitted in that case [64]. So, any denoising/filtering technique is not employed on the raw information in our study. Finally, the major failure case of our proposed method is the inability to identify all categories of images correctly available in real worlds including the identification of all beat images properly, which is demonstrated in Figures 5(a), 6(a), 8, and 9 and Tables 9 and 10. However, 2D CNN-based deep method is a promising direction for diagnosing various categories of cardiovascular diseases in offline and online approaches.

## 4. Conclusions

In this study, a 2D CNN method with an effective DenseNet is proposed for arrhythmias recognition on four different imbalanced datasets with various experiments. The findings from all experiments demonstrate that the proposed method outperforms the performance of state-of-the-art models, which validates the proposed method's effectiveness and generalization. The key convenience of the developed model is that each layer can access the gradients directly from the input signals and loss function, resulting in improved gradients and information flow across the network with various regularization techniques. These regularizing effects alleviate the overfitting challenges on classification tasks with the confined training data sizes. Moreover, our experimental results from all experiments illustrate that the proposed model provides satisfactory results in resolving the class imbalance issue of all used datasets. The findings also indicate that the performance of the developed model remains almost identical despite using various strategies in various experiments for four heterogeneous datasets. This expresses better applicability and scalability of the proposed method. So, the proposed method could be a helpful tool for cardiologists' clinical decision support systems in offline or online approaches. The factors behind such successes are (i) because of using indicated regularization techniques, (ii) advantages of the fundamental DenseNets model compared to others such as features reusing, the punctuation of features propagation, and less trained parameters to be required, (iii) proper segmentation and transformation of beat images, and (iii) because of using weighted categorical cost function and weighted random sampler in all experiments. In the future, we will look into a hybrid model incorporating LSTM with the developed model. We have also planned to conduct a study with the clinical data or data from our developed flexible sensor to test the proposed method, which will be more applicable in real-life applications. It is also possible to employ the study in other biomedical engineering applications, especially in neurological diseases such as Alzheimer's, epilepsy.

## Figures and Tables

**Figure 1:** The workflow of the proposed method (a) with stratified K-fold cross-validation (in case of *E*_3_, *E*_4_, *E*_7_, and *E*_8_, the model is in only evaluation mode); (b) using transfer learning mechanism (in case of *E*_5_, *E*_6_, *E*_9_, and *E*_10_).

**Figure 2:** ECG signal representation such as (a) heartbeat segmentation demonstration, (b) normal beat, (c) supraventricular ectopic beat, (d) ventricular ectopic beat, (e) fusion beat, and (f) unknown beat.

**Figure 3:** The proposed DenseNet model structure with three dense blocks.

**Figure 4:** (a) Internal structure of a dense block, where every convolutional layer receives the outputs from all prior layers as the input, and (b) structure of a transition block.

**Figure 5:** (a) Confusion matrix from MIT-BIH arrhythmia dataset in *E*_1_, and (b) training and testing loss curve for *E*_1_.

**Figure 6:** (a) Confusion matrix from INCART arrhythmia dataset in *E*_2_, and (b) training and testing loss curve for *E*_2_.

**Figure 7:** Graphs for the three matrices such as accuracy, *F*_1-score_, and recall in (a) *E*_1_ and (b) *E*_2_.

**Figure 8:** Reached confusion matrix in (a) *E*_3_ and (b) *E*_4_.

**Figure 9:** Reached confusion matrix in (a) *E*_5_ and (b) *E*_6_.

**Figure 10:** Training and testing loss curve for (a) *E*_5_ and (b) *E*_6_.

**Figure 11:** Training and testing loss curve for (a) *E*_9_ and (b) *E*_10_.

**Table 1:** The developed DenseNet model's internal architecture, including relevant hyperparameters. ReLU, BN, fully connected, and softmax layers are not shown here.

Dense blocks	Layers name	Output size	Kernel size	# Filters	Stride	Padding
Primary convolution layer	Conv2d-1	128 × 128	7 × 7	64	2	3

Dense_Block-1	Conv2d-4	128 × 128	3 × 3	32	1	1
	Conv2d-6	128 × 128	3 × 3	32	1	1
	Conv2d-9	128 × 128	3 × 3	32	1	1
	Conv2d-12	128 × 128	3 × 3	32	1	1
	Conv2d-15	128 × 128	3 × 3	32	1	1

Transition layer -1	Conv2d-19	128 × 128	1 × 1	128	1	0
	AvgPool2d-22	64 × 64	2 × 2	128	2	0

Dense_Block-2	Conv2d-25	64 × 64	3 × 3	32	1	1
	Conv2d-27	64 × 64	3 × 3	32	1	1
	Conv2d-30	64 × 64	3 × 3	32	1	1
	Conv2d-33	64 × 64	3 × 3	32	1	1
	Conv2d-36	64 × 64	3 × 3	32	1	1

Transition layer -2	Conv2d-40	64 × 64	1 × 1	128	1	0
	AvgPool2d-43	32 × 32	2 × 2	128	2	0

Dense_Block-3	Conv2d-46	32 × 32	3 × 3	32	1	1
	Conv2d-48	32 × 32	3 × 3	32	1	1
	Conv2d-51	32 × 32	3 × 3	32	1	1
	Conv2d-54	32 × 32	3 × 3	32	1	1
	Conv2d-57	32 × 32	3 × 3	32	1	1

Transition layer -3	Conv2d-61	32 × 32	1 × 1	64	1	0
	AvgPool2d-64	16 × 16	2 × 2	64	2	0

**Table 2:** A summary of metrics from confusion matrix depicted in Figure 5(a).

Accuracy(%)		Precision (%)		Recall (%)		*F *_1score_ (%)	
N	99.81	N	99.97	N	99.82	N	99.90
S	99.96	S	99.08	S	99.45	S	99.26
V	99.86	V	98.32	V	99.73	V	99.02
F	99.97	F	95.53	F	99.52	F	97.49
Average	99.90	Average	98.23	Average	99.63	Average	98.92

**Table 3:** A summary of metrics from confusion matrix depicted in Figure 6(a).

Accuracy (%)		Precision (%)		Recall (%)		*F *_1score_ (%)	
N	99.63	N	99.96	N	99.64	N	99.80
S	99.98	S	99.53	S	98.42	S	98.97
V	99.65	V	95.60	V	99.63	V	97.57
F	99.99	F	99.07	F	100.0	F	99.53
Average	99.81	Average	98.54	Average	99.42	Average	98.97

**Table 4:** The comparison of all evaluation metrics and validation loss for both experiments.

Evaluation matrices/validation loss	*E *_1_	*E *_2_
Recall	0.9963	0.9942
*F *_1-score_	0.9891	0.9891
Accuracy	0.9980	0.9963
Precision	0.9834	0.9894
Minimal validation loss	0.0233	0.0234

**Table 5:** A summary of all evaluated metrics from confusion matrix depicted in Figures 8(a) and 8(b).

Accuracy (%)		Precision (%)		Recall (%)		*F *_1score_ (%)	
*For E *_3_							
N	99.70	N	100.0	N	99.69	N	99.85
S	100.0	S	100.0	S	100.0	S	100.0
V	100.0	V	100.0	V	100.0	V	100.0
F	99.70	F	75.00	F	100.0	F	85.71
Average	99.85	Average	93.75	Average	99.92	Average	96.39

*For E *_4_							
N	99.94	N	100.0	N	99.94	N	99.97
S	100.0	S	100.0	S	100.0	S	100.0
V	100.0	V	100.0	V	100.0	V	100.0
F	99.94	F	93.75	F	100.0	F	96.77
Average	99.97	Average	98.44	Average	99.98	Average	99.19

**Table 6:** The comparison of all reached metrics in *E*_3_ and *E*_4_.

Evaluation matrices	*E *_3_	*E *_4_
Recall	0.9992	0.9998
*F *_1-score_	0.9639	0.9919
Accuracy	0.9970	0.9994
Precision	0.9375	0.9844

**Table 7:** A summary of all evaluated metrics from confusion matrix depicted in Figures 9(a) and 9(b).

Accuracy(%)		Precision (%)		Recall (%)		*F *_1score_ (%)	
*For E *_5_							
N	99.67	N	99.90	N	99.79	N	99.84
S	99.67	S	94.46	S	97.28	S	95.85
V	100.0	V	100.0	V	100.0	V	100.0
F	100.0	F	100.0	F	100.0	F	100.0
Average	99.83	Average	98.59	Average	99.27	Average	98.92

*For E *_6_							
N	99.87	N	99.96	N	99.90	N	99.93
S	99.87	S	97.59	S	98.91	S	98.25
V	100.0	V	100.0	V	100.0	V	100.0
F	100.0	F	100.0	F	100.0	F	100.0
Average	99.94	Average	99.39	Average	99.70	Average	99.55

**Table 8:** The comparison of all reached metrics in *E*_5_ and *E*_6_.

Evaluation matrices/validation loss	*E *_5_	*E *_6_
Recall	0.9927	0.9971
*F *_1-score_	0.9892	0.9954
Accuracy	0.9970	0.9987
Precision	0.9859	0.9939
Minimal validation loss	0.0236	0.0236

**Table 9:** The reached confusion matrix and average values of evaluated metrics in *E*_7_ and *E*_8_.

	Predicted label					Accuracy (%)	Precision (%)	Recall (%)	*F *_1_score_ (%)
		F	N	S	V				
*E *_7_									
True label	F	62	0	0	1	99.92	95.27	98.03	96.62
	N	0	10585	10	0				
	S	4	0	75	0				
	V	0	1	0	90				

*E *_8_									
True label	F	62	0	1	0	99.94	97.41	98.68	98.03
	N	0	10590	5	0				
	S	2	0	77	0				
	V	0	1	0	90				

**Table 10:** The reached confusion matrix and average values of evaluated metrics in *E*_9_ and *E*_10_.

	Predicted label					Accuracy (%)	Precision (%)	Recall (%)	*F *_1_score_ (%)
		F	N	S	V				
*E *_7_									
True label	F	119	0	0	2	99.89	97.37	99.15	98.38
	N	2	43500	10	4				
	S	0	0	166	2				
	V	0	2	0	362				

*E *_8_									
True label	F	120	0	0	1	99.98	98.51	99.58	99.03
	N	1	43506	6	3				
	S	0	1	167	0				
	V	0	0	1	363				

**Table 11:** Comparative table of our work with the previous approaches.

Classifier type/approach	Class categories	Accuracy	Precision	Recall	*F*1-score
2D CNN (proposed) (on MIT-BIH-E_1_)	4	99.80^*∗∗*^	98.34^*∗∗*^	99.63^*∗∗*^	98.91^*∗∗*^
2D CNN (proposed) (on INCART-E_2_)	4	99.63^*∗∗*^	98.94^*∗∗*^	99.42^*∗∗*^	98.91^*∗∗*^
2D CNN [36]	8	98.92^*∗*^	—	97.26^*∗*^	98.00^*∗*^
		99.11^*∗∗*^	—	97.91^*∗∗*^	98.00^*∗∗*^
2D CNN [39]	8	99.05^*∗*^	—	97.85^*∗*^	—
		98.90^*∗∗*^	—	97.20^*∗∗*^	
2D CNN [39] AlexNet	8	98.85^*∗*^	—	97.08^*∗*^	—
		98.81^*∗∗*^	—	96.81^*∗∗*^	
2D CNN [39] VGGNet	8	98.63^*∗*^	—	96.93^*∗*^	—
		98.77^*∗∗*^	—	97.26^*∗∗*^	
2D CNN [37]	4	98.50^*∗*^	—	—	—
2D CNN [38]	8	99.02^*∗∗*^	—	—	—
2D CNN [58]	5	99.00^*∗*^	—	—	—
2D CNN [59]	5	99.70^*∗∗*^	—	99.70^*∗∗*^	—
2D CNN [60]	5	99.62^*∗*^	—	92.24^*∗*^	94.00^*∗*^
1D CNN [36]	8	97.80^*∗*^	—	—	—
1D CNN [58]	5	90.93^*∗*^	—	—	—
1D CNN [38]	5	97.38^*∗*^	—	—	—
CNN-LSTM [61]	5	98.10^*∗*^	—	97.50^*∗*^	—
LSTM, FL [62]	8	99.26^*∗*^	—	99.26^*∗*^	—
DBB, AdaBoost [12]	5	99.10^*∗*^	—	97.90^*∗*^	—

^*∗∗*^with augmentation on-the-fly or manual, ^*∗*^without augmentation, FL: focal loss, DBB: distribution-based balancing.

## Data Availability

The data used to support the findings of the study are available from the Mr. Hadaate Ullah (hadaate@std.uestc.edu.cn) upon request.

## References

[1] Keidar N., Elul Y., Schuster A., Yaniv Y. (2021). Visualizing and quantifying irregular heart rate irregularities to identify atrial fibrillation events. *Frontiers in Physiology*.

[2] Malik S. A., Parah S. A., Malik B. A. (2022). Power line noise and baseline wander removal from ECG signals using empirical mode decomposition and lifting wavelet transform technique. *Health Technology*.

[3] Bock C., Kovacs P., Laguna P., Meier J., Huemer M. (2021). Ecg beat representation and delineation by means of variable projection. *IEEE Transactions on Biomedical Engineering*.

[4] Lee M., Lee J. H. (2022). A robust fusion algorithm of LBP and IMF with recursive feature elimination-based ECG processing for QRS and arrhythmia detection. *Applied Intelligence*.

[5] Saxena S., Vijay R., Saxena G., Pahadiya P. (2022). Classification of cardiac signals with automated R-peak detection using wavelet transform method. *Wireless Personal Communications*.

[6] Chandrasekar A., Shekar D. D., Hiremath A. C., Chemmangat K. (2022). Detection of arrhythmia from electrocardiogram signals using a novel Gaussian assisted signal smoothing and pattern recognition. *Biomedical Signal Processing and Control*.

[7] Alfaras M., Soriano M. C., Ortin S. (2019). A fast machine learning model for ECG-based heartbeat classification and arrhythmia detection. *Frontiers in Physiology*.

[8] Bhattacharyya S., Majumder S., Debnath P., Chanda M. (2021). Arrhythmic heartbeat classification using ensemble of random forest and support vector machine algorithm. *IEEE Transaction. Artificial. Intelligent.*.

[9] Lai D., Heyat M. B. B., Khan F. I., Zhang Y. (2019). Prognosis of sleep bruxism using power spectral density approach applied on EEG signal of both EMG1-EMG2 and ECG1-ECG2 channels. *IEEE Access*.

[10] Heyat M. B. B., Lai D., Khan F. I., Zhang Y. (2019). Sleep bruxism detection using decision tree method by the combination of C4-P4 and C4-A1 channels of scalp EEG. *IEEE Access*.

[11] Acharya U. R., Oh S. L., Hagiwara Y. (2017). A deep convolutional neural network model to classify heartbeats. *Computers in Biology and Medicine*.

[12] Rajesh K. N. V. P. S., Dhuli R. (2018). Classification of imbalanced ECG beats using re-sampling techniques and AdaBoost ensemble classifier. *Biomedical Signal Processing and Control*.

[13] Iqbal M. S., Abbasi R., Bin Heyat M. B. (2022). Recognition of mRNA N4 acetylcytidine (ac4C) by using non-deep vs. Deep learning. *Applied Sciences*.

[14] Yan W., Zhang Z. (2021). Online automatic diagnosis system of cardiac arrhythmias based on MIT-BIH ECG database. *Journal of Healthcare Engineering*.

[15] Teelhawod B. N., Akhtar F., Heyat M. B. B. Machine learning in E-health: a comprehensive survey of anxiety.

[16] Akhtar F., Heyat M. B. B., Li J. P., Patel P. K., Guragai B. Role of machine learning in human stress: a review.

[17] Hannun A. Y., Rajpurkar P., Haghpanahi M. (2019). Cardiologist-level arrhythmia detection and classification in ambulatory electrocardiograms using a deep neural network. *Nat. Med.*.

[18] Lyu S., Liu J. (2021). Convolutional recurrent neural networks for text classification. *Journal of Database Management*.

[19] Ullah H., Bin Heyat M. B., AlSalman H. (2022). An effective and lightweight deep electrocardiography arrhythmia recognition model using novel special and native structural regularization techniques on cardiac signal. *Journal of Healthcare Engineering*.

[20] Yildirim Ö. (2018). A novel wavelet sequence based on deep bidirectional LSTM network model for ECG signal classification. *Computers in Biology and Medicine*.

[21] Chen C., Hua Z., Zhang R., Liu G., Wen W. (2020). Automated arrhythmia classification based on a combination network of CNN and LSTM. *Biomedical Signal Processing and Control*.

[22] Guragai B. A survey on deep learning classification algorithms for motor imagery.

[23] Muaad A. Y., Jayappa H., Al-antari M. A., Lee S. (2021). ArCAR: a novel deep learning computer-aided recognition for character-level Arabic text representation and recognition. *Algorithms*.

[24] Bin Heyat B., Hasan Y. M., Siddiqui M. M. (2015). EEG signals and wireless transfer of EEG Signals. *Int. J. Adv. Res. Comput. Commun. Eng.*.

[25] Algarni M., Saeed F., Al-Hadhrami T., Ghabban F., Al-Sarem M. (2022). Deep learning-based approach for emotion recognition using electroencephalography (EEG) signals using Bi-directional long short-term memory (Bi-LSTM). *Sensors*.

[26] Heyat M. B. B., Akhtar F., Azad S. (2016). Comparative analysis of original wave and filtered wave of EEG signal used in the prognostic of bruxism medical sleep syndrome. *International Journal of Trend in Scientific Research and Development*.

[27] AlShorman O., Masadeh M., Heyat M. B. B. (2022). Frontal lobe real-time EEG analysis using machine learning techniques for mental stress detection. *Journal of Integrative Neuroscience*.

[28] Heyat M. B. B., Akhtar F., Khan M. H. (2021). Detection, treatment planning, and genetic predisposition of bruxism: a systematic mapping process and network visualization technique. *CNS & Neurological Disorders - Drug Targets*.

[29] El Gannour O., Hamida S., Cherradi B. (2021). Concatenation of pre-trained convolutional neural networks for enhanced covid-19 screening using transfer learning technique. *Electronics*.

[30] Akhtar F., Patel P. K., Heyat M. B. B. (2022). Smartphone addiction among students and its harmful effects on mental health, oxidative stress, and neurodegeneration towards future modulation of anti-addiction therapies: a comprehensive survey based on slr, Research questions, and network visualization techniques. *CNS & Neurological Disorders - Drug Targets*.

[31] Bin Heyat M. B., Akhtar F., Khan A. (2020). A novel hybrid machine learning classification for the detection of bruxism patients using physiological signals. *Applied Sciences*.

[32] Ullah H., Bu Y., Pan T. Cardiac arrhythmia recognition using transfer learning with a pre-trained DenseNet.

[33] Weimann K., Conrad T. O. F. (2021). Transfer learning for ECG classification. *Scientific Reports*.

[34] He K., Zhang X., Ren S., Sun J. Deep residual learning for image recognition.

[35] Huang G., Liu Z., Van Der Maaten L., Weinberger K. Q. Densely connected convolutional networks.

[36] Ullah A., Anwar S. M., Bilal M., Mehmood R. M. (2020). Classification of arrhythmia by using deep learning with 2-D ECG spectral image representation. *Remote Sensing*.

[37] Xu P., Liu H., Xie X., Zhou S., Shu M., Wang Y. (2022). Interpatient ECG arrhythmia detection by residual attention CNN. *Computational and Mathematical Methods in Medicine*.

[38] Ullah A., Rehman S.S., Mehmood R. M.M. (2021). A hybrid deep CNN model for abnormal arrhythmia detection based on cardiac ECG signal. *Sensors*.

[39] Jun T. J., Nguyen H. M., Kang D., Kim D., Kim D., Kim Y. H. (2018). ECG Arrhythmia Classification Using a 2-D Convolutional Neural Network. http://arxiv.org/abs/1804.06812.

[40] Rubin J., Parvaneh S., Rahman A., Conroy B., Babaeizadeh S. (2018). Densely connected convolutional networks for detection of atrial fibrillation from short single-lead ECG recordings. *Journal of Electrocardiology*.

[41] Al Rahhal M. M., Bazi Y., Almubarak H., Alajlan N., Al Zuair M. (2019). Dense convolutional networks with focal loss and image generation for electrocardiogram classification. *IEEE Access*.

[42] Lin T. Y., Goyal P., Girshick R., He K., Dollar P. (2020). Focal loss for dense object detection. *IEEE Transactions on Pattern Analysis and Machine Intelligence*.

[43] Du C., Liu P. X., Zheng M. (2022). Classification of imbalanced electrocardiosignal data using convolutional neural network. *Computer Methods and Programs in Biomedicine*.

[44] Fernando K. R. M., Tsokos C. P. (2022). Dynamically weighted balanced loss: class imbalanced learning and confidence calibration of deep neural networks. *IEEE Transactions on Neural Networks and Learning Systems*.

[45] Ioffe S., Szegedy C. Batch normalization: accelerating deep network training by reducing internal covariate shift.

[46] Garatti S., Campi M. C. (2022). Complexity is an effective observable to tune early stopping in scenario optimization. *IEEE Transactions on Automatic Control*.

[47] Shekelyan M., Cormode G., Triantafillou P., Shanghooshabad A., Ma Q. (2022). Weighted Random Sampling over Joins. https://arxiv.org/pdf/2201.02670.pdf.

[48] Kingma D. P., Ba J. L. Adam: A Method for Stochastic Optimization.

[49] Lam T. K., Ohta M., Schamoni S., Riezler S. (2021). On-the-fly aligned data augmentation for sequence-to-sequence ASR. *Interspeech 2021*.

[50] He K., Zhang X., Ren S., Sun J. Delving deep into rectifiers: surpassing human-level performance on imagenet classification.

[51] Ghorbani Afkhami R., Azarnia G., Tinati M. A. (2016). Cardiac arrhythmia classification using statistical and mixture modeling features of ECG signals. *Pattern Recognition Letters*.

[52] Muaad A. Y., Jayappa Davanagere H., Benifa J. V. B. (2022). Artificial intelligence-based approach for misogyny and sarcasm detection from Arabic texts. *Computational Intelligence and Neuroscience*.

[53] Jahin D., Emu I. J., Akter S., Patwary M. J., Bhuiyan M. A. S., Miraz M. H. A novel oversampling technique to solve class imbalance problem: a case study of students’ grades evaluation.

[54] Nawabi A. K., Jinfang S., Abbasi R. (2022). Segmentation of drug-treated cell image and mitochondrial-oxidative stress using deep convolutional neural network. *Oxidative Medicine and Cellular Longevity*.

[55] Bin Heyat M. B., Akhtar F., Abbas S. J. (2022). Wearable flexible Electronics based cardiac electrode for researcher mental stress detection system using machine learning models on single lead electrocardiogram signal. *Biosensors*.

[56] Sultana A., Rahman K., Heyat M. B. B., Sumbul, Akhtar F., Muaad A. Y. (2022). Role of inflammation, oxidative stress, and mitochondrial changes in premenstrual psychosomatic behavioral symptoms with anti-inflammatory, antioxidant herbs, and nutritional supplements. *Oxidative Medicine and Cellular Longevity*.

[57] Chen D., Li D., Xu X., Yang R., Ng S. K. (2021). Electrocardiogram classification and visual diagnosis of atrial fibrillation with DenseECG. https://arxiv.org/abs/2101.07535.

[58] Huang J., Chen B., Yao B., He W. (2019). ECG arrhythmia classification using STFT-based spectrogram and convolutional neural network. *IEEE Access*.

[59] Degirmenci M., Ozdemir M. A., Izci E., Akan A. (2021). Arrhythmic Heartbeat Classification Using 2D Convolutional Neural Networks. *Irbm*.

[60] Zhang Y., Li J., Wei S., Zhou F., Li D. (2021). Heartbeats classification using hybrid time-frequency analysis and transfer learning based on ResNet. *IEEE Journal of Biomedical and Health Informatics*.

[61] Oh S. L., Ng E. Y., Tan R. S., Acharya U. R. (2018). Automated diagnosis of arrhythmia using combination of CNN and LSTM techniques with variable length heart beats. *Computers in Biology and Medicine*.

[62] Gao J., Zhang H., Lu P., Wang Z. (2019). An effective LSTM recurrent network to detect arrhythmia on imbalanced ECG dataset. *Journal of Healthcare Engineering*.

[63] Dinakarrao S. M. P., Jantsch A., Shafique M. (2020). Computer-aided arrhythmia diagnosis with bio-signal processing: a survey of trends and techniques. *ACM Computing Surveys*.

[64] Andersen R. S., Peimankar A., Puthusserypady S. (2019). A deep learning approach for real-time detection of atrial fibrillation. *Expert Systems with Applications*.

